The article "Analysis on the Influence of Students' Health Quality Based on Intelligent Optimization of Sports Facilities and Equipment" was retracted in 2023. Reasons: signs of a paper mill; suspected computer-generated content; unreliable results or conclusions; lack of ethics approval or compliance.

# Analysis on the Influence of Students' Health Quality Based on Intelligent Optimization of Sports Facilities and Equipment

**DOI:** 10.1155/2022/8145127

**Published:** 2022-01-15

**Authors:** Qi Zhou

**Affiliations:** School of Physical Education, Shandong Normal University, Jinan, Shandong 250014, China

## Abstract

Physical health promotion has always been a way for schools to pay close attention to and devote resources to their students' development, physical fitness, and social adaptability. To promote the improvement of students' overall physical quality, we must begin with the foundation and school physical education. This study proposes an improved K-means algorithm based on an analysis of the influencing factors of intelligent optimization of sports facilities and equipment on students' health quality. Clustering analysis is carried out based on two groups of data classified as boys and girls, using the improved K-means algorithm. The findings reveal that the average change trend of physical fitness test items in each male cluster is generally similar, with a moderate change. The change in the average score of physical fitness test items for each cluster of girls in the group showed two distinct valleys, and the trend was complicated. This necessitates schools to invest funds to construct venues and purchase equipment in order to increase the number of sporting events.

## 1. Introduction

As an important part of school education, school physical education is an effective way to improve quality education. It can lay a solid foundation for crazy sports, competitive sports, and lifelong sports and plays an important role in promoting students' health [1]. Sports venue equipment is the basic objective condition of school physical education. Whether the venue equipment is ready to be perfected is the key for teachers to achieve teaching objectives and tasks, and whether the venues and equipment can be reasonably used is an important link to improve teaching quality [2, 3]. The venue is the material guarantee implemented by the physical education class. Without the venue, physical education class will not be able to do it. Without the equipment or equipment shortage, it will not only affect the physical education class but also make students feel bored and reduce their enthusiasm so that physical education class cannot normally do it and cannot achieve the expected effect. Sports venue equipment plays a vital role in school sports [4].

The concept of school education is critical for college students' development [5]. The form, content, and innovative teaching methods of physical education are critical to the development of university physical education in the university curriculum. Currently, there are numerous issues with the construction of sports facilities and equipment, and numerous nuances in the intelligent design of competition venues. The design scheme is mixed up with the intelligent construction of other facilities during construction, causing the specific construction to become disorganized, and changing the construction scheme also delays the construction period and the use effect [6, 7]. In our country's university sports facilities, there are currently some issues, such as a lack of intelligent sports services, unscientific management, and a low level of openness and sharing [8]. As a result, if the country promotes the wide adoption of the internet of things and the development of the sports internet of things, these issues can be solved one by one using the technologies, concepts, and functions of the internet of things.

The article "Analysis on the Influence of Students' Health Quality Based on Intelligent Optimization of Sports Facilities and Equipment" was retracted in 2023. Reasons: signs of a paper mill; suspected computer-generated content; unreliable results or conclusions; lack of ethics approval or compliance.

By understanding students' physical health problems, it is found that students get more physical exercises in their study and life, constantly improve their own health, face life and study with a healthier body, and develop comprehensive moral, intellectual, and physical qualities. Therefore, this study not only embodies the concrete practical significance but also has certain theoretical value [9]. This study tries to find out the factors that affect students' health quality by investigating the intelligent optimization of sports facilities and equipment. So as to put forward some constructive suggestions, students' health quality should be improved, and a little contribution should be made to the school's physical education.

At present, the number of college students is increasing. Faced with a large number of student data, it is difficult for teachers to design personalized exercise prescriptions for each student, so as to efficiently and scientifically improve students' physical quality. Therefore, it is the focus of this study to use reasonable methods to analyze and evaluate physical test data and reasonably classify students, and how to reasonably recommend prescriptions. In order to solve the above problems, data mining technology is applied to cluster analysis of data samples by the K-L-Hearts algorithm. According to the characteristics of clustering results, some suggestions for improving physical fitness are put forward.

## 2. Related Work

According to literature [10] through the investigation of some schools, it is found that there is little difference in the quantity, compliance, and usage of essential sports equipment among schools of different sizes. Literature [11] mentioned that the investment in sports funds was insufficient; the number of students in the school is increasing year by year, which leads to the shortage of sports facilities in the school; due to the development of cities, land use is particularly tight; schools lack specialized sports management and maintenance personnel: the degree of socialization is not enough; school leaders do not pay enough attention to sports. Literature [12, 13] point out that the development of school sports cannot be separated from the management of school sports equipment protection and maintenance, which is extremely important. Literature [14–16] found that schools only pay attention to the construction of sports venues that occupy a small area, are easy to carry out sports events, are popular with popular students, have many functions, and have low investment costs. Literature [17] found that as long as sports venues and facilities' equipment are geared toward competitive sports, the degree of openness of sports facilities in schools is not enough, and students are charged for the use of some expensive facilities. The emergence of some problems is related to the development of present sports.

The article "Analysis on the Influence of Students' Health Quality Based on Intelligent Optimization of Sports Facilities and Equipment" was retracted in 2023. Reasons: signs of a paper mill; suspected computer-generated content; unreliable results or conclusions; lack of ethics approval or compliance.

According to literature [18], from the relationship between sports and nutrition, it is discussed that the abnormal phenomenon that most of the quality development levels show a downward trend is closely related to the reduction in physical exercise and extracurricular activities caused by students' heavy learning burden. Literature [19] suggests that aiming at the increase in obesity among students, on the basis of strengthening students' exercise, also publicizes the impact of various food intake on physical fitness and regularly arranges strict physical examination; literature [20] concludes that malnutrition rate, especially severe malnutrition rate, is obviously decreasing, while overweight and obesity rates are increasing, so teenagers should have a reasonable diet, watch less TV, play less computer, strengthen physical exercise, and increase outdoor activities in their spare time. Literature [21] discusses that the reasons for examination-oriented education system, society, and family should pay for the decline of students' physical health. The comparison of before and after improvements in physical fitness test indicators in the literature [22] reveals a lack of health awareness among school leaders and teachers, and sports health has not been elevated to the highest or most important goal of student development. According to the literature [23], senior students are overweight or underweight. Despite the fact that the student's test scores were mostly passing, the excellent rate and the good rate are low, indicating that the student's physical health is not promising. The physical health of female college students was investigated in the literature [24], which discovered and analyzed the differences in physical health between different types of students. [25] According to a survey of college students from various regions of China, there are differences in physical fitness among college students. Shorter students in the Western region have poorer physical fitness, while taller students in the Eastern region have better physical functions.

The article "Analysis on the Influence of Students' Health Quality Based on Intelligent Optimization of Sports Facilities and Equipment" was retracted in 2023. Reasons: signs of a paper mill; suspected computer-generated content; unreliable results or conclusions; lack of ethics approval or compliance.

## 3. Research Method

### 3.1. Health Overview

Physical health is our most concerned topic. There is a close relationship between physical fitness and health, and they are highly similar in terms of “good health.” Usually, people with good health have healthy bodies, and people with healthy bodies also have good health. But this statement is not absolute, and there are differences in meaning between them.

When evaluating the health and physique of individuals, there are also differences in measurement and evaluation techniques and standards. When evaluating the physique of individuals, the first thing to think about is the health status and then the inductive evaluation of their shape, function, physical quality, sports strength, and psychology.

In order to improve students' physical health, we must first find ways to increase their awareness of physical activity and cultivate healthy sports attitudes. We all know that one of the factors affecting students' physical health is their lack of awareness of physical exercise, so it is critical to increase their awareness of physical exercise. As we all know, the body is the foundation of learning, and scientific and effective physical exercise is the best way for us to get healthy and learn.

Every student is an individual, and their ability to receive education and their ability to receive physical education differ. PE teachers should develop corresponding teaching plans based on individual student characteristics and teach students according to their aptitude when teaching courses, in order to more quickly promote the healthy development of students' physiques. Physical education teachers should make accurate assessments of students' strengths based on their current circumstances so that students can better showcase their own strengths, address any weaknesses, and boost their self-confidence.

### 3.2. Intelligent Optimization of Sports Equipment and Facilities

In the twenty-first century, the social competitive pressure is becoming more and more intense. It not only includes superficial intellectual competition but also tests on physical and psychological aspects. These nonintellectual factors determine the success or failure of competition at the same time, and the important factor that determines this aspect is the health status. However, at present, some groups of college students lack the awareness of exercising, and their awareness of exercising is scientifically weak. Therefore, it is the key to effectively and scientifically improve college students' health quality, and exercise prescription is the best way to effectively and scientifically improve their health.

The article "Analysis on the Influence of Students' Health Quality Based on Intelligent Optimization of Sports Facilities and Equipment" was retracted in 2023. Reasons: signs of a paper mill; suspected computer-generated content; unreliable results or conclusions; lack of ethics approval or compliance.

Whether or not the sports facilities and equipment are perfect will have a significant impact not only on teaching but also on the improvement of national competitive sports. Imperfect sports venues and facilities and a lack of good venues and equipment will not pique students' interest in sports learning, limiting their active participation in physical activity and limiting their physical quality improvement. Because they lack adequate venues and equipment, some students become bored with physical education classes. It is possible that they are uninterested, in which case their grades will not improve. Independent modules are used to create dependent modules. Independent modules can determine the built positions of other independent modules by creating and solving models. Dependent modules should be grouped together with the independent modules on which they rely. The model can be established as follows.

Assume that the dependent module *X*_*m*_ depends on the independent module *X*_1_, *X*_2_,…, *X*_*a*_; *m*=*n*_1_+1,…, *n*, *a*=*n*_1_. Then, the mathematical model with the least cost for establishing the dependent module is as follows:

(1) $$\begin{array}{c} \min\sum_{i=1}^{a}f_{mi}d_{mi}. \end{array}$$

The secondary facility planning method is adopted. First, all facilities are sorted in order of importance and area, and the ones with larger importance and area are taken out as independent modules. In this example, the first 8 modules are divided into independent modules and the next 25 modules are divided into dependent modules. The optimized layout model of independent modules is established as follows:

(2) $$\begin{array}{c} \min\sum_{i=1}^{8}\sum_{j=1}^{8}\sum_{k=1}^{8}\sum_{l=1}^{8}C_{ijkl}X_{ik}X_{jl}. \end{array}$$

When the module *i* is built in position *k*, it is *x*_*ik*_=1, and otherwise, it is 0. The distance matrix between locations is *D*, and the transportation matrix between modules is *F*. It is required that these eight facility modules must be built at these eight locations to minimize the total cost.

After the independent module is optimized, a simple mathematical model is established for the remaining 25 dependent modules, assuming that the dependent module *X*_*m*_ depends on the independent module *X*_1_, *X*_2_,…, *X*_8_; *m*=9,…, 33. Then, the mathematical model with the least cost for establishing the dependent module is as follows:

(3) $$\begin{array}{c} \min\sum_{i=1}^{8}f_{mi}\sqrt{{\left(x_{m}-x_{i}\right)}^{2}={\left(y_{m}-y_{i}\right)}^{2}}. \end{array}$$

The development balance of school teaching projects is linked to the irrational allocation of sports equipment. *M* schools only allocate some sports venues with low costs, multiple functions, and less land occupation, preventing some sports events from taking place; the single content of physical education in schools leads to unbalanced development of teaching items, while the allocation of school sports equipment is solely based on teaching items. Due to a slew of issues, sports facilities are being allocated in an irrational manner. The lack of attention given to school physical education by schools and educational authorities is the primary cause of these phenomena.

The article "Analysis on the Influence of Students' Health Quality Based on Intelligent Optimization of Sports Facilities and Equipment" was retracted in 2023. Reasons: signs of a paper mill; suspected computer-generated content; unreliable results or conclusions; lack of ethics approval or compliance.

### 3.3. Analysis of College Students' Physical Health

The massive data and powerful analytical abilities of big data will provide more valuable possibilities for the promotion of students' physical health in concept and how to reveal hidden, previously unknown, and potentially practical information from the massive fuzzy and noisy historical data of practical application databases. The goal of clustering analysis is to group things into classes based on some attributes, with the as little similarity between classes as possible and as much similarity within classes as possible.

Clustering analysis is to reasonably divide data, establish classification according to certain principles, and determine the existence of data category by analyzing each record of original data in a historical record database. If the data sample set under study is *M*, *C* is defined as a nonempty subset of a sample set *M*: *C* ⊂ *M* and *C* ≠ ∅. Clustering is to satisfy the following conditions under the set of class *C*_1_, *C*_2_,…, *C*_*k*_:

(4) $$\begin{array}{c} \left\{\begin{array}{c} C_{1}\cup C_{2}\cup \cdots C_{k}=M,\\ C_{i}\cap C_{j}=\emptyset . \end{array}\right. \end{array}$$

According to the first condition, each sample in the sample set *M* has a class corresponding to it, while the second condition indicates that each sample of *M* belongs to at most one class.

K-means algorithm is a typical distance-based clustering algorithm, which uses distance as the evaluation criterion of similarity, that is, the closer the distance between two objects, the greater the similarity. It can well solve the clustering problem of numerical attribute data objects. The algorithm is as follows:

1. Randomly select *k* records from *n* records as centroid
2. Measure each remaining record, get its distance to each centroid, and classify it to the nearest centroid class
3. Recalculate the obtained centroid of each class

Iterate for 2 ∼ 3 steps until the new centroid is equal to the original centroid or less than the specified threshold; then, the algorithm ends.

The article "Analysis on the Influence of Students' Health Quality Based on Intelligent Optimization of Sports Facilities and Equipment" was retracted in 2023. Reasons: signs of a paper mill; suspected computer-generated content; unreliable results or conclusions; lack of ethics approval or compliance.

The flow of the K-means clustering algorithm is shown in Figure 1.

K-means is widely used because of its simplicity and easy realization. However, this algorithm has some defects. In this section, we will propose an improved algorithm to optimize the K-means algorithm.

The distance is calculated from each cluster center to other cluster centers, and half of the minimum distance is expressed as *d*_*e*(*i*)_, that is, half of the minimum distance from the *i* th cluster center to other cluster centers. For all data points, the distance to the *i* th cluster center is calculated and compared with *d*_*e*(*i*)_, respectively.

If the distance is less than or equal to *d*_*e*(*i*)_, the data point is assigned to the *i* th cluster; otherwise, the distance from the point to other cluster centers is calculated. This process is repeated until the data point is assigned to other clusters. If the data point cannot be assigned to any cluster, it is put in the cluster where the nearest cluster center is located.

The improved algorithm is as follows:

(5) $$\begin{array}{c} d_{e\left(i\right)}=\frac{\min\left\{\left|C_{i},C_{j}\right|\right\}}{2}, \end{array}$$

where *d*_*e*(*i*)_ is 1/2 of the minimum distance from the *i* th cluster to other clusters.

(6) $$\begin{array}{c} d\left(Z_{p},M_{j}\right)=\sqrt{\sum_{k=1}^{d}{\left(Z_{p,k}-M_{j,k}\right)}^{2}}, \end{array}$$

where *Z*_*p*_ is the *p* -th data point, *M*_*j*_ is the centroid of the *j* -th cluster, and *d* is the dimension.

(7) $$\begin{array}{c} M_{j}=\frac{1}{n_{j}}\left(\sum_{\nabla Z_{p}\in C_{j}}Z_{p}\right), \end{array}$$

where *n*_*j*_ is the number of data points in the cluster *j*.

According to the requirements of the K-means algorithm, SPSS Modeler software is used to design clustering models for the records of boys and girls, respectively, as shown in Figure 2.

For male students, seven fields including vital capacity score, 50 m score, 1,000 m score, standing long jump score, sitting body flexion score, pull-up score, and total score are selected as input fields. For girls, seven fields, namely, vital capacity score, 50 m score, 800 m score, standing long jump score, sitting body flexion score, one-minute sit-up score, and total score, are selected as input fields.

After clustering, the results are divided into 1–5 categories. The larger the average score in these 5 categories of data, the better the students' sports performance in this index. Then, this value can be used to compare the same items in five types of data and analyze the running model to obtain clustering results.

The article "Analysis on the Influence of Students' Health Quality Based on Intelligent Optimization of Sports Facilities and Equipment" was retracted in 2023. Reasons: signs of a paper mill; suspected computer-generated content; unreliable results or conclusions; lack of ethics approval or compliance.

## 4. Result Analysis and Discussion

### 4.1. Analysis on the Demand of Sports Venues and Equipment and Students' Participation in Sports Activities

Sporting activities are a way for students to unwind during their free time. The development of sports activities not only helps to relieve brain fatigue, but it also helps to relax the tense mood of the day, which is beneficial to students' health and has an impact on their physical fitness. Currently, all of the district's schools offer sports activities, but the majority of them focus on running, which distorts the concept of sports. The reason for this is that sports facilities are not sufficiently equipped to meet the needs of students.

After-school sports training is an effective means to cultivate students' hobbies, improve sports skills, and train talents for the country. It provides the source power for the development of school sports, is also an important part of China's current sports training system and mechanism, and is the foundation of cultivating outstanding sports talents in China.

Sports training needs to be based on sports venues and equipment. Sufficient sports venues and equipment can better tap their own potential and improve their own quality and skill level.  Figure 3 shows the demand analysis of sports venue equipment and after-school sports practice.

Through the questionnaire survey of teachers, 60% of physical education teachers think that they cannot meet the needs of extracurricular physical education training, and 8% even think that they are not satisfied. Through interviews with teachers, the shortage of school sports facilities also directly affects students' training plans, and some students are particularly interested in emerging sports programs. However, due to the lack of sports facilities, such sports programs cannot be developed, which restricts the provision of sports reserve talents.

After a series of sports interventions, the subjects were retested, and it was found that the students' test scores were significantly improved. From the comparison before and after (Figure 4), the excellent rate and good rate of the test were significantly improved, especially the good rate increased by 10 percentage points, and the passing rate of the students was also decreasing. On the whole, the average scores of the students were effectively improved. Therefore, reasonable and scientific physical exercise can obviously improve students' physical quality.

The article "Analysis on the Influence of Students' Health Quality Based on Intelligent Optimization of Sports Facilities and Equipment" was retracted in 2023. Reasons: signs of a paper mill; suspected computer-generated content; unreliable results or conclusions; lack of ethics approval or compliance.

Boys' test scores are steadily improving, as evidenced by the results of girls' tests (Figure 5). Girls' scores also have noticeable improvement. Girls' test pass rate has increased to 100% following the sports intervention, and the excellent and good rates are also improving. The data of the subjects are constantly improving in the above tests of boys and girls, and the effect is visible when students are subjected to aerobic exercises such as variable speed running and endurance running. As a result, students must engage in relevant scientific physical exercises on a regular basis in order to improve their cardiopulmonary function.

### 4.2. Analysis of Students' Health Quality

#### 4.2.1. Analysis of K-Means Clustering Algorithm

Experiments will prove that the improved K-means algorithm improves the accuracy of clustering and reduces the number of iterations. In this study, Iris, wine, balance, and Pima data from the UCI database are selected as experimental data. The experimental hardware environment is Intel (*R*) Pentium (*R*) dual-core CPU 2.2 GHz, 2 GB memory, and 1 50G hard disk. The environment is Windows XP operating system, MATLAB.

Figure 6 is the experimental result of the average running average accuracy obtained by executing the two algorithms 100 times for these four datasets, respectively.

From this figure, the improved algorithm avoids the unreasonable division caused by randomness when the original algorithm selects the initial clustering center by selecting the part of the data object set as the initial clustering center. So that the data point objects can be divided into more reasonable clusters. Therefore, the average accuracy of classification can be effectively improved.

Figure 7 is the experimental result of the average running time obtained by executing the two algorithms 100 times for these four datasets, respectively.

From this figure, it can be seen that the improved algorithm first improves the selection of the initial clustering center, thus reducing the running time of the algorithm. Second, because the traditional K-means algorithm needs to calculate the distance between data points and each cluster, the improved algorithm only needs to calculate the distance between data points and one cluster in the best case, so the average running time of the improved algorithm is significantly less than that of the original algorithm.

#### 4.2.2. Results Analysis of Clustering

After summarizing the average scores of each individual physical quality of five types of students in the boys' group and girls' group, it can be seen that each cluster has its own characteristics. The results of clustering and the specific analysis of each cluster are as follows.

1. The clustering results of boys are shown in Figure 8.
2. The average total score of each item of cluster 1 boys is the highest and that of cluster 3 boys is the lowest. In 50 m, 1,000 m, standing long jump, sitting forward, and pull-ups, students in cluster 1 scored the highest, while students in cluster 3 scored the lowest except pull-ups. Students in cluster 5 of vital capacity items scored the highest.
3. Cluster students also have the lowest score; there is little difference between the pull-up scores of boys in cluster 1 and cluster 4, but the pull-up scores of boys in clusters 2, 3, and 5 are extremely poor, especially the average pull-up scores of boys in cluster 2 are in single digits. Generally speaking, the pull-up scores of boys in five categories are the lowest, which also reflects the serious shortage of boys' upper limb strength.
4. The 50 m, 1,000 m, sitting posture flexion, and pull-up of clustered boys have excellent performances among the five types of students, and the average of these four scores ranks second.

The article "Analysis on the Influence of Students' Health Quality Based on Intelligent Optimization of Sports Facilities and Equipment" was retracted in 2023. Reasons: signs of a paper mill; suspected computer-generated content; unreliable results or conclusions; lack of ethics approval or compliance.

Compared with the results of boys' clustering, the change in average scores of different items in each cluster of girls is more complicated. The average scores of girls after clustering are shown in Figure 9.

Cluster 1, 3, and 4 girls' scores of each item have the same changing trend, while cluster 2 and cluster 5 have great contrast between each item. The average score of cluster 1 in the listed seven items is far higher than that of other clusters, and the number of records occupied by cluster *L* is the highest. The average score of vital capacity of cluster 3 girls is only 10.12, and the average score of sitting body flexion of cluster 5 girls is 18.96, forming two abnormally prominent valleys.

The average total scores of girls in cluster 3 and cluster 5 rank first and second from the bottom, respectively, due to the large differences in these two items' scores. Cluster 2 girls have the lowest scores in the 50 m, 800 m, standing long jump, and sit-ups, but there is little difference between them and the other four clusters, so they are in the middle of the average total score comparison. The change trend of clustered girls' scores eased and remained high, while the average scores of all other scores ranked second, except for 800 m and sit-ups.

### 4.3. Suggestion

Relevant leaders of the Education Bureau and schools should attach importance to the development of school sports, increase investment in sports facility construction, and equip a set of perfect sports equipment for students to use. The school should be regularly supervised and inspected, especially the sports field equipment, and the school should be urged to strengthen the construction of sports field equipment. To establish a standardized sports equipment room, there should be explicit regulations and requirements for the entrance and exit of equipment. In the absence of sports venues and equipment, the diversity of site and equipment use should be known.

The article "Analysis on the Influence of Students' Health Quality Based on Intelligent Optimization of Sports Facilities and Equipment" was retracted in 2023. Reasons: signs of a paper mill; suspected computer-generated content; unreliable results or conclusions; lack of ethics approval or compliance.

Schools should be people-oriented and meet the needs of students participating in sports activities; as a result, stadiums and facilities must be quickly built, and funds must be invested to purchase appropriate sports equipment. Physical education teachers should use this as a foundation for vigorously developing sports, enriching students' enjoyment of sports activities, allowing more students to participate in sports activities, enriching students' sports lives, and promoting students' athletic development. Physical health tests for students are not only a school requirement but also a good opportunity for students to learn about their physical condition. Students should have a clear and comprehensive understanding of their own physical information and the issues that come with it. The cause should be determined in light of the issue. For example, some common issues in girls include a severe lack of lower limb strength, poor aerobic exercise ability, and boys' weak upper limb strength, among others. When choosing sports events, all types of students should consider improving their physical quality with weak or serious information displays.

To deeply analyze the physique information of physique measurement data, not only the data from the horizontal direction is analyzed, but also the physique information of many years is compared vertically, and the regularity of its presentation is explored, so as to effectively predict the physique quality, which is in the trend of inferior development. From a scientific point of view, it is far from enough to only investigate the status quo of physical health. The reasons for the status quo of physical information should be deeply analyzed, effective intervention to the actual status should be made, and feedback information should be collect in real time to adjust and improve the intervention measures in time to fundamentally solve the actual problems.

## 5. Conclusions

There is a significant disparity between the school's physical education courses and students' preferred sports, preventing students from improving their physical fitness and mastering their skills. Due to the influence of sports facilities, some sports cannot be offered, resulting in students' lack of enthusiasm for physical education class. Overall, the subject test data are unsatisfactory, and the scores are on the verge of passing. There are few samples with noticeable data, particularly in boys' pull-ups, and many subjects fail the test. Clustering results show that there are obvious deficiencies in upper and lower limb strength levels of male and female students, respectively, based on the overall trend. As a result, it is necessary to investigate the internal relationship between students' physical fitness and indicators based on clustering results in order to promote physical health and in order to significantly improve students' physical health.

The article "Analysis on the Influence of Students' Health Quality Based on Intelligent Optimization of Sports Facilities and Equipment" was retracted in 2023. Reasons: signs of a paper mill; suspected computer-generated content; unreliable results or conclusions; lack of ethics approval or compliance.

The algorithm's time complexity and performance need to be improved further. The improved algorithm will easily degenerate into the traditional K-means algorithm in the worst case or when the amount of data is small, so the next step is to improve the algorithm for these two special cases.

## Figures and Tables

**Figure 1:** Algorithm flowchart.

**Figure 2:** K-means clustering model.

**Figure 3:** Analysis of the demand for sports venue equipment and after-school sports practice in mainland China.

**Figure 4:** Comparison of male students' vital capacity test.

**Figure 5:** Comparison of girl's vital capacity test.

**Figure 6:** Hundred times average running average accuracy experimental results.

**Figure 7:** Experimental result chart of 100 times average running time.

**Figure 8:** Change trend of average scores of boys after clustering.

**Figure 9:** Change trend of average scores of girls after clustering.

## Data Availability

The data used to support the findings of this study are included within the article.

## References

[1] Giménez-Meseguer J., Tortosa-Martínez J. (2021). The influence of physical condition on mental health and quality of life in patients with drug dependence. *Journal of Addictions Nursing*.

[2] Mozolev O., Shorobura I., Zdanevych L., Hutsal L., Marusynets M., Kravchuk L. (2020). Influence of physical fitness of students on the quality of leisure organization in a sports and health tourism. *Revista Romaneasca pentru Educatie Multidimensionala*.

[3] Muhammad R., Dara Hanifa R. (2019). The influence of health promotion on female students’’ behaviour in SMA an - nizam medan about endometriosis. *Open access Macedonian journal of medical sciences*.

[4] Lera-López F., Ollo-López A., Sánchez-Santos J. M. (2017). How does physical activity make you feel better? The mediational role of perceived health. *Applied Research in Quality of Life*.

[5] Kim K. W., Wallander J. L., Peskin M., Cuccaro P., Elliott M. N., Schuster M. A. (2019). Associations between parental SES and children’s health-related quality of life: the role of objective and subjective social status. *Journal of Pediatric Psychology*.

The article "Analysis on the Influence of Students' Health Quality Based on Intelligent Optimization of Sports Facilities and Equipment" was retracted in 2023. Reasons: signs of a paper mill; suspected computer-generated content; unreliable results or conclusions; lack of ethics approval or compliance.

[6] Wang R. (2019). Research on the impact of campus football on the development of pupils’ physical and mental health. *Good day*.

[7] Zeng R., Ye Y., Wu X. (2020). An empirical study of physical fitness training intervention on the physical fitness of primary school students under the background of “Healthy China”. *Journal of Changsha University*.

[8] Wang S. (2019). Analysis and countermeasures of the physical fitness and health status of junior middle school students. *Tomorrow*.

[9] Li X. (2019). Analysis of factors affecting students’’ physical health and reasonable intervention measures. *Friends of Health*.

[10] Ma Z. (2020). Exploration and intervention strategy of physical health education model for primary and middle school students. *Marriage, Education and Health*.

[11] Wang X., Zhu Y. (2019). An empirical study on the effect of physical education intervention on improving the physical fitness of college students. *Stationery & Sports Products & Technology*.

[12] Zhou H. (2019). Analysis and research on the influence of students’ physical fitness on mental health in higher vocational colleges. *Economic and Technical Cooperation Information*.

[13] Wang Y. (2020). The effect of outreach training on the physical and mental health of junior high school students. *Scientific Consultation*.

[14] Xiong B. (2021). Study on the factors affecting the physical health of primary school students and the countermeasures. *Progress: Teaching and Research*.

[15] Li X. (2020). Research on students’’ physical health problems and new influencing factors. *Elementary Education Forum*.

[16] Yuan Y. (2021). Analysis of the main problems in the physical health testing of college students. *Stationery and Sports Articles and Technology*.

[17] Tian B. (2021). Research on the impact of campus running APP on the health of college students. *Science Popular: Science Education*.

[18] Zheng Z. (2019). Research on the effect of high school physical education teaching on the physical health of students. *Contemporary Family Education*.

[19] Wei W. (2020). An empirical study on the impact of physical training on high school students’ physical fitness under the background of core literacy ——taking 2019 students as an example. *Slam Dunk*.

[20] Li Y., Wang Y. (2021). Research on improving the physical fitness of college students. *Sports-Leisure: Mass Sports*.

[21] Huang B. (2020). Influencing factors and implementation suggestions for senior high school students’ physical fitness test scores. *Contemporary Sports*.

[22] Rui L. (2021). Research on the influence of “integration of inside and outside class” teaching mode on college students’’ physical fitness. *Sports Science and Technology Literature Bulletin*.

The article "Analysis on the Influence of Students' Health Quality Based on Intelligent Optimization of Sports Facilities and Equipment" was retracted in 2023. Reasons: signs of a paper mill; suspected computer-generated content; unreliable results or conclusions; lack of ethics approval or compliance.

[23] Xu Z. (2020). Analysis of the causes of the decline of middle school students’ physical fitness and exploration of countermeasures. *Composition Guidance for Middle School Students*.

[24] Zhang R., Huang J. (2021). Southwest university of science and technology students’’ physical fitness test results analysis and countermeasures. *Contemporary Sports Science and Technology*.

[25] Zhang W. (2019). Discussion on the causes and countermeasures of the physical health test of college students. *intelligence*.

